This article has been retracted.

# Identification of a Novel Ferroptosis Inducer for Gastric Cancer Treatment Using Drug Repurposing Strategy

**DOI:** 10.3389/fmolb.2022.860525

**Published:** 2022-07-04

**Authors:** Jinping Zhang, Meimei Gao, Ying Niu, Jiangang Sun

**Affiliations:** ^1^ Department of Gastroenterology, The First Affiliated Hospital of Zhengzhou University, Zhengzhou, China; ^2^ Henan Key Laboratory of Precision Clinical Pharmacy, The First Affiliated Hospital of Zhengzhou University, Zhengzhou, China; ^3^ Department of Gastrointestinal Surgery, The First Affiliated Hospital of Zhengzhou University, Zhengzhou, China

**Keywords:** gastric cancer, ferroptosis, HC-056456, inducer, small molecules

## Abstract

Gastric cancer remains one of the major contributors to global cancer mortality, although there is no promising target drug in clinics. Hence, the identification of novel targeted drugs for gastric cancer is urgent. As a promising strategy for inducing ferroptosis for gastric cancer treatment, the ferroptosis inducer is a potential drug. Nevertheless, no ferroptosis inducer has entered clinics. So, our purpose was to identify a novel ferroptosis inducer for gastric cancer treatment using a drug repurposing strategy. Firstly, using a drug repurposing strategy with the aid of a commercialized compound library, HC-056456, a small molecule bioactive CatSper channel blocker, was characterized to inhibit the growth of gastric cancer line MGC-803. At the same time, this anti-proliferation effect can be blocked by ferrostatin-1, a ferroptosis inhibitor, indicating that HC-056456 is a ferroptosis inducer. Then, HC-056456 was identified to decrease GSH content via p53/SLC7A11 signaling pathway. Then Fe^2+^ and lipid peroxide were accumulated when cells were exposed to HC-056456. Finally, HC-056456 was found to suppress the growth of gastric cancer cells by increasing p53 and repressing SLC7A11 *in vivo* but not in the presence of ferrostatin-1. In sum, we systematically elucidate that HC-056456 exerts anti-gastric cancer effect by provoking ferroptosis *in vitro* and *in vivo*, suggesting its potential role in gastric cancer treatment.

## Introduction

Gastric cancer (GC) is now the fifth most common malignancy in modern society and ranks third in cancer-related mortality (Jiang et al., 2015; Smyth et al., 2020; Fu et al., 2021). Globally, there are estimated to be more than one million new cases of gastric cancer and nearly 800,000 deaths every year (Sano, 2017; Fu et al., 2021). East Asia, Eastern Europe, and South America are the regions with high incidence and mortality of gastric cancer (Uno, 2019; Smyth et al., 2020). In recent years, comprehensive surgical treatment such as endoscopic resection has good efficacy for early gastric cancer (Japanese Gastric Cancer, 2017). However, the vast majority of patients were diagnosed with advanced stages and often accompanied by peritoneal metastasis and liver metastasis, resulting in short 5-years postoperative survival and poor prognosis (Catenacci et al., 2011; Yue et al., 2019). Besides, first-line small molecule drugs for gastric cancer are still the traditional chemotherapy drugs that have been used for a long time, such as 5-fluorouracil and cisplatin (Wagner et al., 2017). Additionally, only a tiny proportion of patients (HER2 or PD-L1-positive) benefit from immunotherapy (Smyth et al., 2020). Thus, research on more effective targeting treatment strategies for gastric cancer is urgently needed.

Ferroptosis is an iron-dependent cell death with oxidative disturbances and reactive oxygen species accumulation in the intracellular microenvironment, different from apoptosis, necrosis, and autophagy (Dixon et al., 2012). In this process, free ferrous iron (Fe^2+^) accumulation and lipid peroxidation are the vital events to induce ferroptosis. In addition, the expression levels of antioxidant systems (GSH) also decreased (Friedmann Angeli et al., 2014). And ferroptosis is terminated by mitochondrial dysfunction and toxic lipid peroxidation. Additionally, p53, the pervasive tumor suppressor factor, is also involved in this process, and it can downregulate the expression of cystine/glutamate antiporter xCT (also known as SLC7A11), thus provoking ferroptosis (Jiang et al., 2015; Liu et al., 2019; Wang et al., 2019; Magri et al., 2021). Other than these macromolecules, some small molecules can also participate in ferroptosis. Iron chelating agents (e.g., deferoxamine) and lipophilic antioxidants (e.g. vitamin E) have inhibitory effects on ferroptosis (Mou et al., 2019). In addition, ferrostatin-1 (Fer-1), N-Acetyl-l-cysteine (NAC), and deferoxamine (DFO) are well-known ferroptosis inhibitors (Liang et al., 2019; Chen et al., 2021; Ding et al., 2021). Fer-1 inhibits ferroptosis by blocking cystine transport and lipoic acid formation. ROS scavenger NAC can reverse the levels of lipid ROS and block ferroptosis. DFO prevents ferroptosis by reducing iron accumulation. What is noteworthy is that ferroptosis can be induced in cancer cells, such as erastin and RSL3 (Jia et al., 2020). Therefore, triggering ferroptosis is spotlighted as a new opportunity to inhibit tumor growth and proliferation (Angelova et al., 2020; Wang et al., 2020; Xia et al., 2020; Ding et al., 2021). Then, the development of ferroptosis inducers presents an attractive therapeutic strategy for cancer.

As a reverse-effectively CatSper channel blocker (Carlson et al., 2009; Orta et al., 2018; Lissabet et al., 2020), HC-056456 was predicted to bind to the center of the CatSper channel with the aid of molecular docking (Lissabet et al., 2020). It was reported that HC-056456 can reduce the CatSper current to prevent over-activation of permissive cultured sperm cells to induce a loss-of-function phenotype (Carlson et al., 2009) and inhibit HCO_3_^−^-induced activation (Orta et al., 2018). In this process, HC-056456 can slow down the rise of intracellular Na^+^ concentration ([Na^+^]_i_) and prevent Ca^2+^ entry caused by alkaline depolarization. Moreover, the CatSper channel can be activated by extracorpuscular progesterone and prostaglandins (Lishko et al., 2011; Strunker et al., 2011; Miller et al., 2016). But the bioactivity of HC-056456 in cancer remains unexplored.

Here, combined with CCK-8 assay, Fer-1-induced GC cells, and oxidative stress markers, HC-056456 was identified as a novel ferroptosis inducer from Bioactive Compound Library. Subsequently, the underlying mechanisms were revealed. HC-056456 inhibits GC cells *in vitro* and *in vivo*. HC-056456 reduced the expression of p53 and upregulated SLC7A11, strikingly reducing the intracellular GSH, promoting the levels of Fe^2+^, leading to lipid peroxidation accumulation and ferroptosis. Above all, our results highlight the unexplored role of HC-056456 in ferroptosis and thus provide its potential utilization for treating gastric cancer.

## Materials and Methods

### Chemical Libraries

Bioactive Compound Library (L4000), a collection of 4890 Bioactivity compounds, was purchased from TargetMol company, United States, and the purity of the compound is above 98%. All compounds were dissolved to 10 mM using DMSO, and 20 μL of the solution was arranged in a 96-well plate. For the following validation mechanism, HC-056456 was also purchased from TargetMol (United States) individually with a purity of 99.6%.

### Cell Culture

Human gastric cancer lines MGC-803, BGC-823, SNU1, and AGS were obtained from the National Collection of Authenticated Cell Cultures (Shanghai, China). Cells were cultured in high glucose Dulbecco’s modified Eagle’s medium (DMEM, Gibco, United States) supplemented with 10% fetal bovine serum (FBS, Invitrogen, United States), 100 μg/ml penicillin, and 100 U/mL streptomycins (Invitrogen, United States). Cells were incubated at 37°C with 5% CO_2_.

### High through-Put Screen

The Cell Counting Kit-8 (CCK-8, Dojindo, Japan) assay was used to measure cell proliferation. MGC-803 cells were seeded in the 96-well plate at a density of 3000 cells per well incubated at 37°C, 5% CO_2_ for 24 h. Then, compounds belonging to the Bioactive Compound Library purchased from TargetMol (United States) were added in the presence of Fer-1 or not, and dimethyl sulphoxide (DMSO) was used as control. After co-incubating for 72 h, 10 μL CCK-8 was added to each well and incubated for 3 h at 37°C. Then the absorbance was measured at 450 nm with a multimode plate reader (PerkinElmer Envision, United States).

### Cell Viability Assay

MGC-803 cells, BGC-823 cells, SNU1 cells, and AGS cells were seeded in the 96-well plate with 3000 cells per well. Then plates were set in a 37°C incubator containing 5% CO_2_ for 24 h. HC-056456, purchased from TargetMol (United States), was added to the medium from 80 μM by 1:1 ratio in the presence of Fer-1 or not, and dimethyl sulphoxide (DMSO) was used as control. After co-incubating for 72 h, 10 μL CCK-8 was added to each well and incubated for 3 h at 37°C. The absorbance was obtained at 450 nm with a multimode plate reader (PerkinElmer Envision, United States). Half inhibitory concentration was calculated by GraphPad Prism 7.0.

### Morphological Changes Analysis

MGC-803 cells were incubated with HC-056456 in the presence of Fer-1 or not. 12 h after incubation, the “ballooning” phenotype was captured by fluorescence microscope at 20× and 40× (Battaglia et al., 2020; Battaglia et al., 2022). 24 h after incubation, the morphological changes were captured by fluorescence microscope at 10×.

### Cell Death Manner Analysis

Gastric cancer cell lines were seeded in the 96-well plate for 24 h. HC-056456 with MGC-803 at 4 μM, BGC-803 or AGS at 10 μM, incubating with necroptosis inhibitor Necrostatin-1 (Necro-1, 10 μM), autophagy inhibitor 3-Methyladenine (3-MA, 2 mM), apoptosis inhibitor Z-VAD-FMK (Z-VAD, 10 μM) and ferroptosis inhibitors N-Acetyl-l-cysteine (NAC, 5 mM), deferoxamine (DFO, 200 μM), and Ferrostatin-1 (Fer-1, 2 μM), independently.

### Lipid Peroxidation Assay

MGC-803 cells were seeded with 6-well plates with 5 × 10^5^ cells/well. After cell adhesion, DMSO, HC-056456 (4 μM), and HC-056456 (4 μM) with Fer-1 (2 μM) were added, respectively. After 8 h incubation, the medium was discarded, and cells were washed with phosphate balanced solution (PBS). Then, C11-BODIPY 581/591 (GLPBIO, United States) was added to the well at a final concentration of 2 μM. The plate was then placed in an incubator at 37°C in 5% CO_2_ for 30 min away from light. After incubation, the fluorescence intensity to assess lipid peroxidation level was analyzed by a fluorescence microscope (T100, Nikon, Japan).

### Western Blot Analysis

MGC-803 cells were collected from 6-well plates, and the lysate was harvested with radioimmunoprecipitation assay (RIPA) buffer containing 1 mM phenylmethylsulfonyl fluoride (PMSF). Cell extracts were quantified by bicinchoninic acid (BCA) quantitation Kit. Protein from each well was separated by 10% sodium dodecyl sulfate-polyacrylamide gel electrophoresis (SDS-PAGE) and transferred to the polyvinylidene fluoride (PVDF) membrane and then blocked with 5% non-fat milk for 2 h. After that, the membrane was co-incubated with the primary antibody at 4°C overnight and followed by incubation with the secondary antibody for 1 h. An enhanced chemiluminescence (ECL) detection kit (Thermo Fisher, United States) was used to check the protein expression.

### Quantitative Real-Time PCR

MGC-803 cells treated with DMSO, HC-056456 (4 μM), and HC-056456 (4 μM) with Fer-1 (2 μM) for 24 h were collected and washed with PBS. RNA was extracted with TRlzol reagent. cDNA was obtained by reverse transcription reaction using PrimeScript™ RT Master Mix kit (Takara, Japan). RT-PCR was carried out by using FastKing-SYBR Green Kit (Tiangen, China). GAPDH Fw 5′-CCA​GCC​GAG​CCA​CAT​CGC-3′, GAPDH Rv 5′-ATG​AGC​CCC​AGC​CTT​CTC​CAT-3′, p53 Fw 5′- ACA​AGG​TTG​ATG​TGA​CCT​GGA-3′, Rv 5′-TGT​AGA​CTC​GTG​AAT​TTC​GCC-3′, SLC7A11 Fw 5′-TCT​CCA​AAG​GAG​GTT​ACC​TGC-3′, SLC7A11 Rv 5′-AGA​CTC​CCC​TCA​GTA​AAG​TGA​C-3′. Data were analyzed by Quantitative Fluorescence PCR (Thermo Fisher, United States).

### Intracellular GSH and Fe^2+^

MGC-803 cells treated with DMSO, HC-056456 (2μM, 4 μM), HC-056456 (2μM, 4 μM) with Fer-1 (2 μM) were collected. Intracellular GSH levels were determined using a glutathione assay kit (Beyotime, China) according to the standard protocol. The quantification of intracellular Fe^2+^ level was carried out using an iron kit (Abcam, UK) according to the manufactory instruction.

### P53 Knockdown

For p53 knockdown, we transduced MGC-803 cells with adenovirus containing a doxycycline-inducible lentiviral shRNA vector. MGC-803 cells were infected with MOI = 10, and the infected cells were selected by culturing monoclonals. Knockdown efficacy was detected by western blot analysis. P53 targeting sequences (Mao et al., 2018; Thiem et al., 2019) were shp53 1# 5′- ACT​CCA​GTG​GTA​ATC​TAC​T-3′, shp53 2# 5′- GTC​CAG​ATG​AAG​CTC​CCA​G-3′, shp53 3# 5′- GACTCCAGT GGTAATCTACT-3′, respectively. A scrambled shRNA was used to serve as a control.

### ADME Evaluation

The molecule structure was drawn and converted into SMILES format by ChemDraw Professional 17.0. SMILES format was inputted to SwissADME online website. Parameters settings such as Lipinski, Ghose, Veber, Egan, and Muegge are displayed on the output web page.

### Prognostic Survival Analysis

SLC7A11 gene expression and clinical survival data were obtained from the TCGA database and the GTEx database, and the correlation between the SLC7A11 expression with tumorigenesis was analyzed by UALCAN (http://ualcan.path.uab.edu/index.html) (Zhou et al., 2022). Kaplan-Meier Plotter was applied to the correlation between patients’ prognosis with SLC7A11 gene expression.

### Nude Mouse Xenograft Models

All animal experiments were approved by the Animal Experiment Ethics Committee of Zhengzhou University. Female BALB/c nude mice aged 4–8 weeks were purchased from Model Animal Research Center, Nanjing University (Nanjing, China). Mice were subcutaneously implanted with 1 × 10^6^ MGC-803 cells under the axilla. The mice were divided into three groups and given orally with vehicle, HC-056456 (50 mg/kg/d), HC-056456 (50 mg/kg/d) and combination with Fer-1 (50 mg/kg/d), respectively. After 14 days, all mice were euthanized, tumor tissues were collected, and tumors were weighed.

### Statistical Analysis

The statistical significance of differences between groups in the *in vitro* study and *in vivo* model was assessed with an unpaired Student’s *t*-test. Results were considered statistically significant at *p* < 0.05. *p* values were displayed on the graphs using a single asterisk for significances ranging from 0.05 to 0.01, two asterisks for values below 0.01, and three asterisks for values below 0.001.

## Results

### HC-056456 Inhibited GC Cells Growth

To find ferroptosis inducers that have therapeutic effects on gastric cancer, compounds from Bioactive Compound Library were screened for their anti-proliferative ability against gastric cancer cell line MGC-803 with the aid of CCK-8 assay and Fer-1 (Figure 1A). The inhibition rate of HC-056456 (Figure 1B) on MGC-803 at 5 μM was 68.1% and could be reversed to 35.6% by Fer-1 (Figure 1C). Then, HC-056456 was verified to have an antiproliferative effect on MGC-803 cells with IC_50_ of 4.32 ± 0.63 μM (Figure 1D), BGC-823 cells with IC_50_ of 6.35 ± 1.53 μM, SNU-1 cells with IC_50_ of 7.34 ± 1.41 μM, and AGS cells IC_50_ of 17.31 ± 1.87 μM (Supplementary Figure S1A-C and Supplementary Table S1). Subsequently, the anti-tumor effect of HC-056456 on MGC-803 cells, BGC-823 cells, SNU-1 cells, and AGS cells was blocked by Fer-1 with IC_50_ of 17.12 ± 1.19 μM (Figure 1E), 20.64 ± 1.31 μM, 18.75 ± 1.62 μM, and 39.33 ± 1.96 μM (Supplementary Figure S1A-C and Supplementary Table S1), respectively. Data demonstrated that HC-056456-induced GC cell growth inhibition was common in gastric cancer. The effect can be offset by Fer-1 to a certain extent.

**FIGURE 1:** HC-056456 exerted anti-proliferation effects on MGC-803, which can be restored by Fer-1 **(A)** Schematic illustration of the procedure of screening promise ferroptosis inducer from Bioactive Compound Library **(B)** Structure of HC-056456 **(C)** The inhibitory rate of HC-056456 (5 μM) on MGC-803 with or without Fer-1 **(D)**The inhibitory effect of HC-056456 on MGC-803. CCK-8 was used to determine the viability of cells **(E)** MGC-803 were exposed to various doses of HC-056456 and Fer-1 (2 μM). Then, CCK-8 was used to determine the viability of cells.

### HC-056456 Induced GC Cells Ferroptosis

To reveal the mechanism of HC-056456, the death manners were analyzed. This experiment used necroptosis inhibitor Necro-1, autophagy inhibitor 3-MA, apoptosis inhibitor Z-VAD, and three known ferroptosis inhibitors, NAC, DFO, and Fer-1. As shown in Figure 2A–C, Supplementary Figures S2A-C and Supplementary Figures S3A-C, compared with HC-056456 treatment, there was no significant change in cell death after combining HC-056456 and Necro-1, 3-MA, and Z-VAD, which indicated that HC-056456 could not induce cell necrosis, autophagy, and apoptosis. Intriguingly, NAC, DFO, and Fer-1 had significant effects on reversing cell death caused by HC-056456 in 3 GC cells (Figure 2D–F, Supplementary Figure S2D-F and Supplementary Figure S3D-F), which suggested that the impact of HC-056456 may be achieved by generating ferroptosis of GC cells. Among the 4 cell lines, MGC-803 had the most noticeable phenotype. And then MGC-803 cell was used as the model in this study.

**FIGURE 2:** The viability of MGC-803 cell lines after the treatment of HC-056456 (10 μM) with **(A)** necroptosis inhibitor Necro-1 (10 μM) **(B)** autophagy inhibitor 3-MA (2 mM) **(C)** apoptosis inhibitor Z-VAD (10 μM) and ferroptosis inhibitors **(D)** NAC (5 mM) **(E)** DFO (200 μM) **(F)** and Fer-1 (2 μM). Results were represented as mean ± SD, **p < 0.01, ***p < 0.001.

### HC-056456 Induced Morphological Changes of MGC-803

Notably, we found that HC-056456 significantly induced morphological changes in MGC-803 cells, while Fer-1 greatly diminished the morphological changes by HC-056456 (Figure 3A). More importantly, “ballooning” was a specific phenotype for ferroptosis cells (Battaglia et al., 2020; Battaglia et al., 2022). Optical microscopy images showed that MGC-803 cells formed the “ballooning” phenotype upon treatment with HC-056456, which can be reversed by Fer-1 (Figure 3B). Taken together, HC-056456 may induce ferroptosis in MGC-803 cells.

**FIGURE 3:** Morphological Changes of MGC-803 **(A)** Optical microscopy images of MGC-803 cells treated with HC-056456 with or without Fer-1 for 24 h (magnification, 10x) **(B)** The “ballooning” phenotype was recorded after HC-056456 treatment for 12 h (magnification, 20x and 40x).

### HC-056456 Promoted Lipid Peroxidation Accumulation

To interrogate this possibility, the effect of HC-056456 on lipid peroxidation accumulation in MGC-803 cells was investigated deeply. Cells treated with HC-056456 in the presence of Fer-1 or not were stained with C11-BODIPY 581/591 and 4’,6-diamidino-2-phenylindole (DAPI) simultaneously and subjected to fluorescence microscope imaging. The results demonstrated that HC-056456 could give rise to the amount of intracellular lipid peroxidation (Figure 4), which can be restored by Fer-1. Together, results indicated that HC-056456 elicits anticancer effects by lipid peroxidation accumulation. All these are in line with ferroptosis.

**FIGURE 4:** HC-056456 induced lipid peroxidation accumulation in MGC-803 cells. MGC-803 cells were treated with vehicle, HC-056456 (4 μM) or HC-056456 (4 μM) in combination with Fer-1 (2 μM) independently for 24 h. The lipid peroxidation was recorded by probe C11-BODIPY 581/591. The photograph was captured by a fluorescence microscope (Scale bar = 50 μm).

### HC-056456 Reduced GSH and Stimulated Fe^2+^ of MGC-803

Then the amount of intracellular GSH and Fe^2+^ were measured. As expected, HC-056456 showed a dose-dependent inhibitory effect on intracellular GSH (Figure 5A). Correspondingly, levels of Fe^2+^ in cells were promoted (Figure 5B). And such signs were hindered when cells were co-incubation with Fer-1. Further exploration of the process was of interest.

**FIGURE 5:** HC-056456 triggered ferroptosis of MGC-803 cells **(A)** The levels of cellular GSH and **(B)** Fe^2+^ were detected. *p < 0.05, **p < 0.01, ***p < 0.001 versus control group.

### HC-056456 Induced Ferroptosis by Regulating P53 and SLC7A11

SLC7A11, essential for glutathione (GSH) synthesis, mainly mediates the uptake of cysteine, which is the vital mechanism for preventing lipid peroxidation and ferroptosis. Additionally, p53 was reported to downregulate SLC7A11 to provoke ferroptosis in cells. To illuminate the mechanism of HC-056456 induced ferroptosis in MGC-803 cells, the expression of SLC7A11 and p53 was detected by western blot and RT-PCR. As Figure 6A–C indicated, HC-056456 dramatically upregulated p53 and repressed SLC7A11 expression. Of note, Fer-1 can alleviate the regulation of HC-056456 on the expression of p53, SLC7A11. To expand our investigation on the mechanism of HC-056456-induced ferroptosis, the p53-knockdown MGC-803 cell line was established by shRNA (Figure 7A). Once p53 was knocked down, the expression of SLC7A11 was significantly increased, and the cell death (Figure 7B) and the intracellular GSH changes induced by HC-056456 were partly blocked (Figure 7C). Interestingly, the reverse effect of Fer-1 on HC-056456 also disappeared. These data suggest that HC-056456 exerted ferroptosis in a p53-dependent manner, resulting in SLC7A11 downregulation and GSH increase.

**FIGURE 6:** HC-056456 enhanced the expression of p53 and downregulated SLC7A11 in MGC-803 cells **(A)** MGC-803 cells were treated as indicated for 24 h. Western Blot detected the expression of p53 and SLC7A11 **(B)** The mRNA levels of p53 and **(C)** SLC7A11 were analyzed by RT-PCR. *p < 0.05, **p < 0.01, ***p < 0.001 versus control group.

**FIGURE 7:** HC-056456 induced ferroptosis in a p53-dependent manner. The p53-knockdown MGC-803 cell was constructed **(A)** The levels of p53 and SLC7A11 were detected by Western Blot **(B)** The viability of cells was calculated **(C)** The level of cellular GSH was carried out. *p < 0.05, **p < 0.01, ***p < 0.001 versus control group.

### ADME Evaluation

SwissADME is a freely available tool in *silico* to evaluate compounds’ druglike properties, including absorption, distribution, metabolism, and excretion, using some predictive rules applied by pharmaceutical chemists (Daina et al., 2017; Brandao et al., 2021). Parameters such as Veber Lipinski and bioavailability can be calculated. Bioavailability radar evaluated that the physicochemical property of HC-056456 is adequate (Figure 8A). Druglikeness predictions showed that HC-056456 meets Lipinski’s rule of five (Figure 8B). The Pharmacokinetics prediction indicated that HC-056456 is more likely the inhibitor of four kinds of CYP and not the substrate of P-gp (Table 1). Boiled-egg model revealed high gastrointestinal absorption of HC-056456 (Figure 8C). All those predict the high oral bioavailability of HC-056456. Combining the bioassays *in vitro* performed in four gastric cancer cell lines, we concluded that HC-056456 could be used as a lead compound for gastric cancer treatment.

**FIGURE 8:** ADME evaluation of HC-056456 was carried out by SwissADME **(A)** Bioavailability radars **(B)** Druglikeness assessment **(C)** Boiled-Egg model assessment.

**TABLE 1:** Pharmacokinetics assessment of HC-056456 as substrate or inhibitor of P-gp or CYP.

Parameters	Pharmacokinetics
P-gp substrate	No
CYP1A2 inhibitor	Yes
CYP2C19 inhibitor	Yes
CYP2C9 inhibitor	Yes
CYP2D6 inhibitor	Yes
CYP3A4 inhibitor	No

### HC-056456 Inhibited Tumor Growth *in Vivo* by Provoking Ferroptosis

Inspired by the anti-tumor effect of HC-056456 *in vitro*, the antitumor activity of HC-056456 *in vivo* was assessed. MGC-803 cells were subcutaneously injected into nude mice to establish the xenograft tumor model (Figure 9A). After 14 days, the tumor volume and weight in mice treated with HC-056456 were significantly smaller than in mice administrated with HC-056456 and Fer-1 simultaneously, indicating the antiproliferative effect of HC-056456 can be partially blocked by Fer-1 (Figure 9B–D). Besides, the intervention did not affect the weight of the mice (Figure 9E). Subsequently, levels of p53 and SLC7A11 in tumors were detected. As expected, the results showed that the HC-056456 up-regulated p53 expression and subsequently down-regulated SLC7a11 *in vivo*, and Fer-1 reversed this effect (Figure 10A,B). The expression of SLC7A11 in gastric cancer in the TCGA database and normal tissue in the GTEx database were analyzed by UALCAN. A statistically significant overexpression in gastric cancer was observed compared with normal tissue (*p* < 0.001, Figure 10C). Concerning prognosis, the expression level of SLC7A11 was negatively correlated with the overall survival (OS, p < 0.001, Figure 10D ), first progression survival (FPS, p < 0.01, Figure 10E ), and post progression survival (PPS, p < 0.001, Figure 10F) of gastric cancer patients, suggesting that SLC7A11 could be a therapeutic target for gastric cancer. Taken together, HC-056456 can inhibit gastric cancer cell growth by inducing ferroptosis *in vivo*.

**FIGURE 9:** HC-056456 inhibited MGC-803 cell growth *in vivo* by inducing ferroptosis in a partially dependent manner **(A)** MGC-803 cells were subcutaneously inoculated in nude mice at a density of 1 × 10^6^. 7 days later (∼100 mm^3^), mice were treated with vehicle, HC-056456 (50 mg/kg/d), HC-056456 (50 mg/kg/d), and Fer-1 (50 mg/kg/d) for 14 days **(B)** Image of tumors was shown after HC-056456 intervention with or without Fer-1 **(C)** Tumor volumes were recorded every 2 days **(D)** Tumors were weighed and recorded **(E)** The weight of mice was monitored. *p < 0.05, **p < 0.01, ***p < 0.001 versus control group.

**FIGURE 10:** HC-056456 excised the anti-gastric cancer effect *in vivo* by upregulating p53 and downregulating SLC7A11 **(A)** The levels of p53 and SLC7A11 of tumors in mice were detected by Western Blot, and **(B)** The pannels were analyzed by ImageJ **(C)** Correlation of SLC7A11 expression between gastric cancer and normal tissues. Relationship between SLC7A11 expression and **(D)** the overall survival **(E)** first progression survival, and **(F)** post progression survival of gastric cancer patients. *p<0.05, **p<0.01, ***p<0.001 versus control group.

## Discussion

Gastric cancer, a malignant tumor with high incidence and mortality rates, remains a considerable risk for health throughout the world (Sexton et al., 2020; Smyth et al., 2020). Surgery is the preferred scheme for patients at an early stage. But most patients are diagnosed at the advanced (or metastatic) stage with a poor prognosis, which overall survival is 10–12 months, and palliative chemotherapy is the primary treatment. Compared with chemotherapy alone, the human epidermal growth factor receptor 2 (HER2) antibody significantly improves the progression-free and overall survival of patients in the first-line treatment (Digklia and Wagner, 2016). But it is limited to patients with HER2 overexpression. On the whole, effective interventions for gastric cancer remain scarce. And the prognosis for patients with advanced gastric cancer remains poor (Patel and Cecchini, 2020). Collectively, research on the novel treatment of gastric cancer is still urgent.

Ferroptosis is a newly discovered type of cell death along with ferrous iron-dependent lipid peroxidation accumulation. And ferroptosis inducers may be a promising strategy for cancer treatment, especially for the eradication of malignancies that are residual or resistant to chemotherapy (Shen et al., 2018; Liang et al., 2019; Mou et al., 2019; Toyokuni et al., 2020). However, few ferroptosis inducers have been reported for gastric cancer (Liu et al., 2021; Mao et al., 2021; Zhao et al., 2021).

In this study, HC-056456 was screened out as a novel ferroptosis inducer from the bioactive compound library. HC-056456 depressed the intracellular GSH and led to Fe^2+^ accumulation. The change of GSH and Fe^2+^ induced a significant increase in lipid peroxidation, thus triggering MGC-803 cells ferroptosis. Especially, HC-056456 exerted the anti-tumor effect in the xenograft tumor model, which can be counteracted by Fer-1. Mechanistically, HC-056456 can upregulate p53 and block system xCT by downregulating SLC7A11 *in vivo* and *in vitro.* Fer-1 can reverse the p53 increase and SLC7A11 block induced by HC-056456. What’s noteworthy is that SLC7A11 is highly expressed in gastric cancer compared with normal tissues. Consistently, high expression of SLC7A11 is associated with a poorer prognosis. These data highlighted the anti-gastric cancer effect of HC-056456.

In summary, this study revealed that HC-056456 can provoke gastric cancer cells ferroptosis *in vitro* and *in vivo*. Taken together, we suggest that HC-056456 can be used as an effective lead compound for the treatment of gastric cancer. And this finding may boost a perspective for ferroptosis inducers in gastric cancer therapeutics.

## Data Availability

The original contributions presented in the study are included in the article/Supplementary Material, further inquiries can be directed to the corresponding author.
